The article "Auxiliary Diagnosis of Lung Cancer with Magnetic Resonance Imaging Data under Deep Learning" was published in 2022. Journal: Comput Math Methods Med.

# Auxiliary Diagnosis of Lung Cancer with Magnetic Resonance Imaging Data under Deep Learning

**DOI:** 10.1155/2022/1994082

**Published:** 2022-05-04

**Authors:** Lei Xia

**Affiliations:** Cancer Center, The Second Affiliated Hospital of Chongqing Medical University, Chongqing 400000, China

## Abstract

This study was aimed at two image segmentation methods of three-dimensional (3D) U-shaped network (U-Net) and multilevel boundary sensing residual U-shaped network (RUNet) and their application values on the auxiliary diagnosis of lung cancer. In this study, on the basis of the 3D U-Net segmentation method, the multilevel boundary sensing RUNet was worked out after optimization. 92 patients with lung cancer were selected, and their clinical data were counted; meanwhile, the lung nodule detection was performed to obtain the segmentation effect under 3D U-Net. The accuracy of 3D U-Net and multilevel boundary sensing RUNet was compared on lung magnetic resonance imaging (MRI) after lung nodule segmentation. Patients with benign lung tumors were taken as controls; the blood immune biochemical indicators progastrin-releasing peptide (pro-CRP), carcinoembryonic antigen (CEA), and neuron-specific enolase (NSE) in patients with malignant lung tumors were analyzed. It was found that the accuracy, sensitivity, and specificity were all greater than 90% under the algorithm-based MRI of benign and malignant tumor patients. Based on the imaging signs for the MRI image of lung nodules, the segmentation effect of the RUNet was clearer than that of the 3D U-Net. In addition, serum levels of pro-CRP, NSE, and CAE in patients with benign lung tumors were 28.9 pg/mL, 12.5 ng/mL, and 10.8 ng/mL, respectively, which were lower than 175.6 pg/mL, 33.6 ng/mL, and 31.9 ng/mL in patients with malignant lung tumors significantly (*P* < 0.05). Thus, the RUNet image segmentation method was better than the 3D U-Net. The pro-CRP, CEA, and NSE could be used as diagnostic indicators for malignant lung tumors.

## 1. Introduction

Primary bronchial lung cancer is referred to lung cancer for short, which is the malignant tumor with the highest mortality in China and in the world. In recent years, with the increase in smokers and the release of harmful gases, the air pollution has been worsening, and both the incidence and mortality of lung cancer have an obvious increasing trend, which seriously influences human health and life. Since 2003, China has promulgated a number of clinical standards for the diagnosis and treatment of tumors, including the *Chinese Guidelines for Diagnosis and Treatment of Primary Lung Cancer* by the Ministry of Health and the *Chinese Version of National Comprehensive Cancer Network* [1–3]. Many researchers have proven that the survival rate of lung cancer patients can be promoted under guideline-based treatment. However, the prognosis of lung cancer patients is still very poor at present. For the high malignancy, relatively difficult treatment, and rapid metastasis, the metastasis of lung cancer has occurred locally or systemically of a considerable part of patients at the time of diagnosis. Generally speaking, the treatment principle of lung cancer is in accordance with multidisciplinary integration treatment and individualized treatment. Common treatment methods in modern medicine include surgery, radiotherapy, chemotherapy, and vaccination [4]. With the continuous update of chemotherapy and radiotherapy protocols and the popularization of new targeted therapies, it is necessary to predict and evaluate the treatment effects of terminal non-small-cell lung cancer (NSCLC). Thereby, the individualized treatment plan can be adjusted as soon as possible to avoid delays by improper treatment, and the prognosis of patients can be improved to the maximum extent [5, 6].

The article "Auxiliary Diagnosis of Lung Cancer with Magnetic Resonance Imaging Data under Deep Learning" was published in 2022. Journal: Comput Math Methods Med.

In recent years, magnetic resonance imaging (MRI) technology has made great progress, such as the high-efficiency gradient imaging technique and parallel imaging technique [7]. The success of these technologies has greatly promoted the application of various lung imaging technologies in clinical diagnosis and treatment. Compared with computed tomography (CT) and positron emission tomography- (PET-) CT, MRI scanning does not have any radioactivity and is therefore safer for patients [8]. The paramagnetic contrast agents that can shorten the time of echo (TE) have been introduced, which enhances the magnetic resonance signal while reducing the susceptibility effect near the cross-area organizational interface [9]. Dynamic contrast-enhanced magnetic resonance imaging (DCE-MRI) can extract a variety of quantitative parameters from the time-intensity curve [10]. These parameters have been proven in numerous clinical studies to be surrogate indicators of tumor diffusion, blood flow, microvessel density, and capillary permeability [11]. Semiquantitative DCE-MRI parameters, like time to peak, maximum enhancement ratio, A, B, C, and D time-intensity signal curves, and pharmacokinetic parameters, have shown the potential to differentiate lung lesions [12]. Studies have shown that DCE-MRI can achieve a diagnostic accuracy of 69-92%, which is comparable to dynamic enhanced CT and PET/CT, but MRI can achieve a higher specificity [13].

Among many machine learning methods, deep learning is derived from neural networks. It is a new higher-performance technology, and its representation of data is often based on learning the combination of low-level features, which is to interpret data through cortex learning inspired by human vision [14–16]. Deep learning models are divided into deep neural network (DNN) models and nonneural network models. DNN models mainly include convolutional neural network, self-encoding, recurrent neural network, etc., and gain remarkable achievements in the fields of computer vision and speech recognition [17, 18]. The image segmentation technologies of three-dimensional (3D) U-shaped network (U-Net) and multilevel boundary sensing residual U-shaped network (RUNet) were applied in this study for lung image segmentation of MRI, and the segmentation results were compared. More methods for cancer diagnosis and examination were provided, and the labor for manual segmentation was saved, which helped to focus on the lesions. Therefore, the application value of MRI image data under the convolutional neural network was discussed in the auxiliary diagnosis of lung cancer, so as to give a theoretical basis and the clinical data for further researches.

The article "Auxiliary Diagnosis of Lung Cancer with Magnetic Resonance Imaging Data under Deep Learning" was published in 2022. Journal: Comput Math Methods Med.

## 2. Methodology

### 2.1. Objects of the Study

In this study, 403 patients with lung nodules or masses were chosen, who underwent thoracic MRI examinations and were diagnosed in the hospital from January 2019 to September 2021. Among these patients, some of them were then excluded, including 86 mild cases, 17 cases with lung cancer, 11 cases with cellular lymphoepithelioma, 2 cases with lymphoma, 3 cases with mucoepidermoid carcinoma, 43 cases with squamous cell carcinoma, 6 cases with unclear pathological diagnosis, and 7 cases with unqualified MRI images. All patients in this study or their authorized families signed the informed consent, and this study had been approved by the medical ethics committee of hospital.

Inclusion criteria were as follows: patients were supposed to be diagnosed with solid lesions occupying the lung space, and the largest diameter of the lesions was ≥10 mm without the treatment of radiotherapy or chemotherapy. The patients had no cerebral tissue disease and no history of serious physical trauma (mainly referring to the trauma in the parts directly connected to the nerves, like the spine). The patients had no contraindication to MRI scanning and could cooperate to complete the routine procedure of thoracic MRI scanning. After MRI, surgical resection, and puncture or biopsy, they were not diagnosed with ecological gene cancer through a simple bronchofiberscope examination. Finally, they had the unbroken relevant clinical data.

Exclusion criteria were as follows: patients had contraindications to MRI examination, such as pacemakers, heart valves, aneurysm clips, and metal or other unattached implants. The patients had poor qualitied scanning images with obvious respiratory motion artifacts or magnetic susceptibility artifacts. The patients had other pathologies of primary cancer and severe heart, lung, liver, and kidney dysfunctions, and those were or were suspected of being pregnant or breastfeeding.

The article "Auxiliary Diagnosis of Lung Cancer with Magnetic Resonance Imaging Data under Deep Learning" was published in 2022. Journal: Comput Math Methods Med.

### 2.2. Image Segmentation Algorithm under 3D U-Net

The segmentation network generally needed to be connected to a two-classification network for the determination whether the detected lesion was a real lesion. Classification networks such as Visual Geometry Group 3D, residual network 3D, and Inception 3D were available, with their own advantages. The fully connected Visual Geometry Group layer network solved the issue of gradient disappearance and network degradation through regularization and 3 × 3 × 3 convolution, while residual network shortcut connection could also handle this. The Inception had several filters of different sizes, which reduced the number of tuning parameters required by the network. The specific process of cerebral tissue image segmentation based on the 3D U-Net algorithm is shown in Figure 1.

The U-Net segmentation method is one of the backbones of the medical image segmentation algorithm. The low-level functions and high-level semantic information were fused through the algorithm, and the multiscale information could be better used. These advantages came from its structure of the encoder and decoder and its connection through layer skipping. The original loss function used in this structure was the pixel-level cross-entropy loss function, which could sort each pixel value in the image. Since the pixel sample imbalance was often encountered when segmenting medical CT images, sometimes the loss used included Dice loss, weight cross entropy, and so on. The most commonly used Dice loss is expressed as

(1) $$\begin{array}{c} \text{Dice}=\frac{2\left|Y1\cap Y2\right|}{\left|Y1\right|+\left|Y2\right|}, \end{array}$$

(2) $$\begin{array}{c} \text{Loss}=1-\text{Dice}. \end{array}$$

To deal with the pixel sample imbalance, the generalized Dice loss function was set and defined as

(3) $$\begin{array}{c} \text{GDL}=1-2\frac{\sum_{m=1}^{2}w_{m}\sum_{n}b\;m_{n}qm_{n}}{\sum_{m=1}^{2}w_{m}\sum_{n}b\;m_{n+}qm_{n}}. \end{array}$$

*b* *m*_*n*_ represented the real value of the *l*-st category at the *n*-th pixel, *qm*_*n*_ was the predicted value, and *w*_*m*_ was the weight of each category. Then, the weight *w*_*m*_ was described as

(4) $$\begin{array}{c} w_{m}=\frac{1}{{\left(\sum_{m=1}^{n}b\;m_{n}\right)}^{2}}. \end{array}$$

In addition to the loss, the loss of sensitivity and specificity was computed as

(5) $$\begin{array}{c} \text{Sensitivity}=\frac{\text{AB}}{\text{AB}+\text{EF}}, \end{array}$$

(6) $$\begin{array}{c} \text{Specificity}=\frac{\text{AF}}{\text{AF}+\text{EB}}, \end{array}$$

(7) $$\begin{array}{c} \text{Loss}=\alpha \frac{\sum_{m=1}^{n}{\left(b_{n}-q_{n}\right)}^{2}}{\sum_{m=1}^{n}b_{n}+\beta }+\left(1-\alpha \right)\frac{\sum_{m=1}^{n}{\left(b_{n}-q_{n}\right)}^{2}}{\sum_{m=1}^{n}\left(1-b_{n}\right)+\beta }. \end{array}$$

AB in equation (5) meant the test result was a real sample, and in fact, it was a real sample; EF meant the test result was a negative sample, and it was a negative sample actually. EB in equation (6) meant the test result was a real sample, but it was actually a negative sample; AF meant the test result was a negative sample, but it was a formal sample in fact. *α* balanced the sensitivity and specificity, and *β* was used to handle the situation where certain data was empty and the divisor was 0, *b*_*n*_ was the true value, and *q*_*n*_ was the predicted value.

The article "Auxiliary Diagnosis of Lung Cancer with Magnetic Resonance Imaging Data under Deep Learning" was published in 2022. Journal: Comput Math Methods Med.

For the unbalanced samples, focal loss could also be used. It was expressed as

(8) $$\begin{array}{c} D_{mi}=\left(\log x,x1=1\right). \end{array}$$

### 2.3. RUNet Segmentation Algorithm under Multilevel Boundary Sensing

RUNet is a part of the segmentation network based on the U-Net structure. The difference from U-Net was that it adopted the method of adding feature layer elements on the symmetric oversampling layer, which restored the spatial information of original image as much as possible during the upsampling process. The residual idea was also applied on certain hierarchical blocks. The feature layer of the input layer after the strategy convolution calculation was computed by adding the first and last feature maps, which improved the computational efficiency of backpropagation. The local information and deep global information were combined, as the residual network elements were added. The characteristic equation of the residual calculation process was described as

(9) $$\begin{array}{c} \text{FM}=X+F\left(X\right). \end{array}$$

There was the same feature channel for each feature extraction layer, and the size of the convolution kernel was set as 3 × 3. After each convolutional layer, batch normalization and regularization were performed to optimize the parameters, and finally, the performance of the model was improved. The second part of the boundary detection network was used for the learning and calculation of the boundary between the tumor and the surrounding tissues. Then, the softmax function was used for the probability value of the boundary Release. Finally, the last end-to-end segmentation of the network target area and the boundary detection targets was carried out, and the boundary constraint function was introduced into the loss function, so that the network can be constrained.

(10) $$\begin{array}{c} L\left(xi,yi,zi,f,w,\alpha ,\beta \right)=\alpha \times \text{Lossseg}+\beta \times \text{Loss}=\alpha \times \beta \times \sum \left[\text{zilog}\left(\overset{´}{zi}\right)Ni=1+\left(1-zi\right)\log\left(1-zi\right)\right]. \end{array}$$

In equation (10), *xi* ∈ *Rh* × *l* represented the prostate image; *yi*, *zi* ∈ *Rh* × *l* represented the segmentation prediction label and actual label of the prostate image, respectively; *h* was the height and width of the image, which represented the hyperparameters used to balance the weight of the loss function; and *N* was the total number of the samples, which was the parameter of the model to be solved.

The article "Auxiliary Diagnosis of Lung Cancer with Magnetic Resonance Imaging Data under Deep Learning" was published in 2022. Journal: Comput Math Methods Med.

The similarity coefficients in the segmentation were used to evaluate the difference between the predicted segmentation and the actual segmentation. The limitation was realized through the cross-entropy calculation. The specific process of image segmentation is shown in Figure 2.

### 2.4. MRI Scanning Protocols

1.5 T MR scanners were used. The coils were the 8-channel cardiac array coils, with electrocardiogram triggering as well as respiration compensation during smooth respiration. Precontrast MRI scanning included T1-weighted and T2-weighted imaging in the transverse plane. The pulse-gated T1-weighted fast spin echo images (time of repetition (TR)/TE = 800 ms/8 ms; matrix: 320 × 160) and respiratory-gated T2-weighted fast spin echo images (TR/TE = 7100‐9236 ms/90‐110 ms; matrix: 320 × 224) were acquired within a range of 41 cm in both length and width. The acquired slice thickness was 5 mm, and the slice interval was 1 mm. The scanning area covered that from the thoracic inlet to the adrenal glands.

### 2.5. Lesion Segmentation

Ubuntu16.04 was used as the program running environment, python was the programming language, and keras was the deep learning framework. SimpleITK and PyDicom were installed, which were for the reading of mhd and dicom files, respectively, and then, these files were converted into npy format files to facilitate training.

With the images of the RUNet and 3D U-Net, the open-source ITK-SNAP software was operated for manual drawing and segmentation of the lesion layer by layer as well as the placement of the region of interest along the edge of the lesion. The selected area included the entire tumor without the visible air area. The region of interest in the lesion was manually segmented by two doctors with 5 years or more experience, and the unified results of the two were picked.

The article "Auxiliary Diagnosis of Lung Cancer with Magnetic Resonance Imaging Data under Deep Learning" was published in 2022. Journal: Comput Math Methods Med.

### 2.6. Observation Indicators and Standards

The general data and the imaging sign indicators of 92 patients with lung cancer were counted, and the imaging signs included the lobe where the tumor was located, the largest diameter of the tumor, the lobulation, the spiculation, and the pleural depression. With the benign tumor patients taken as the control group (*n* = 10), blood samples were collected from the patients in two groups. After the serum was separated, the progastrin-releasing peptide (pro-CRP), neuron-specific enolase (NSE), and carcinoembryonic antigen (CEA) in the serum were detected by the enzyme-linked immunosorbent assay.

### 2.7. Statistical Analysis

SPSS Statistics 25.0 was used for the analysis of the clinical data and MRI imaging signs of the 92 patients. The enumeration data was expressed by frequency, the measurement data was expressed by the average value, and the difference comparison was analyzed through the independent sample *t*-test. It was considered to be statistically significant as *P* < 0.05.

## 3. Results

### 3.1. Results of the 3D U-Net Segmentation Algorithm

The LKDS and Luna16 lung nodule detection data sets were utilized for model training, and the acquired MRI images of lung cancer patients were used to verify the model. According to the detection probability worked out by the algorithm, the average FROC value can be calculated. When segmenting the images of lung nodules, different results would be obtained as the different loss function networks were applied. Focal loss was applied to segment lung nodule images at last. Compared with focal loss, Dice loss was not easy to converge. The average value of Dice in the final segmentation was 0.62.

### 3.2. Comparison Results of MRI Lung Nodule Segmentation Algorithms

For the original lung MRI images, the lung nodule areas were segmented under the 3D U-Net and the multilevel boundary sensing RUNet optimized in this study (the red area in Figure 3). The segmented images are shown in Figure 3. It could be observed that the optimized multilevel boundary sensing RUNet had a better performance to segment different lung nodules from the lung MRI image more clearly and completely.

### 3.3. Evaluation of Image Segmentation Results

Quantitative analysis and comparison were carried out for the evaluation indicators including true positive (TP), false positive (FP), false negative (FN), Jaccard similarity (JS), accuracy, sensitivity, and specificity. These quantitative statistical indicators of benign and malignant tumors were compared and analyzed, as shown in Figures 4 and 5. From these quantitative indicators, both the two segmentation algorithms had good segmentation performance. The RUNet model had a TP of 81 and a JS of 79% for diagnosis of benign tumors, as well as a TP of 82 and a JS of 79.5% for diagnosing malignant tumors; the specificity and sensitivity were better than those of the 3D U-Net model.

The article "Auxiliary Diagnosis of Lung Cancer with Magnetic Resonance Imaging Data under Deep Learning" was published in 2022. Journal: Comput Math Methods Med.

### 3.4. Test Results of Biochemical Indicators of Lung Cancer Patients

The differences of pro-CRP, NSE, and CAE in serum between benign and malignant lung cancer patients are shown in Figure 6. It was observed that the pro-CRP, NSE, and CAE in the serum of patients with malignant lung tumors were 175.6 pg/mL, 33.6 ng/mL, and 31.9 ng/mL, respectively, while those of patients with benign lung tumors were 28.9 pg/mL, 12.5 ng/mL, and 10.8 ng/mL, respectively. After comparison, it was found that serum levels of pro-CRP, NSE, and CAE of patients with malignant lung tumors were significantly higher than those of patients with benign lung tumors (*P* < 0.05).

## 4. Discussion

There are still many shortcomings in the U-Net model; for example, the extraction effect of boundary edges in medical image segmentation is particularly unsatisfactory. To deal with the shortcomings of the U-Net, the multilevel boundary sensing RUNet model was proposed. The network structure in the RUNet was composed of the segmentation network based on the U-Net structure and the network multilevel boundary detection. End-to-end training and learning were supplemented into the same network structure, as segmentation and boundary positioning were realized [19, 20]. The jumper connection strategy is widely used in U-Net, residual net, and dense net. By this method, not only was the information conversion cross layer between networks improved but also more spatial image information was restored during the oversampling process. Thereby, the network gradient disappearance was solved, and a deeper network structure was achieved [21, 22]. Thus, the residual jumper connection method was applied for gradient disappearance caused by too deep network layers. In the lesion identification in MRI images of lung cancer patients under deep learning algorithms, it was found that the diagnostic sensitivity of the RUNet is significantly higher than that of the 3D U-Net, but the recognition accuracy and specificity of 3D U-Net are better than those of the RUNet. The difficulty of lung contour segmentation was that there would be a great difference of the area ratio of two connected areas, as sometimes there were two lungs in one connection area, but the second connection area showed nothing when the images were processed under the 3D U-Net.

MRI examination has a high clinical application value for identifying benign and malignant lung lesions. MRI has no ionizing radiation and can be repeated for several times in a short period, with great safety. An inversion recovery echo diffusion sequence is used. On the basis of the fact that the background signals of the tissue (muscle, fat, liver, etc.) are fully suppressed, the diffusion-weighted contrast between the lesion area and the surrounding tissue is more prominent. Thereby, the ability to distinguish the tumor tissue from the surrounding tissue is improved. While the RUNet was used in 5lung MRI image processing, cross-multilevel boundary could be perceived more clearly, and it was easier to distinguish two connected areas. Therefore, the RUNet was more convenient and efficient in multilevel boundary detection.

The article "Auxiliary Diagnosis of Lung Cancer with Magnetic Resonance Imaging Data under Deep Learning" was published in 2022. Journal: Comput Math Methods Med.

In addition to imaging data, serum-oncologic indicators are often used in the diagnosis of cancer. Both pro-CRP and CEA are autonomous growth factors for the treatment of small-cell lung cancer [23]. Studies have shown that the expression level of CEA in the digestive tract, breast, lung, and other tissues of patients with malignant tumors is significantly increased [24]. NSE is a type of glycoprotein mainly in nerve tissues. It has been often used in the diagnosis of tumors, and some studies suggest that the expression level of NSE in lung cancer patients is 10 times that of normal tissues [25]. In this study, the pro-CRP, CEA, and NSE in the serum of patients with malignant and benign tumors were detected and compared. The results demonstrated that all the levels of pro-CRP, CEA, and NSE in malignant lung tumor patients increased significantly, which suggested that these indicators can be used as biochemical indicators for the diagnosis of malignant lung tumors.

## 5. Conclusion

This study was made to explore the application value of the 3D U-Net and multilevel boundary sensing RUNet segmentation methods in auxiliary diagnosis of lung cancer with lung MRI image data. The results showed that the multilevel boundary sensing RUNet gained a clearer image effect than the 3D U-Net for MRI image segmentation of lung nodules. Besides, the blood immune biochemical indicators of pro-CRP, CEA, and NSE were significantly higher in malignant lung tumor patients. This study was single-centered, the sample size was small, and there was no external verification of the model, all of which were the shortcomings. In the further studies in the future, multicenter trials with larger sample size should be carried out and verified. As the samples will increase, the clarity of lung MRI images under the two segmentation methods will also be compared further in depth, so that the research foundation and clinical data for the diagnosis of lung cancer would be enriched.

The article "Auxiliary Diagnosis of Lung Cancer with Magnetic Resonance Imaging Data under Deep Learning" was published in 2022. Journal: Comput Math Methods Med.

## Figures and Tables

**Figure 1:** The flowchart of the 3D U-Net image segmentation algorithm.

**Figure 2:** Flowchart of the multilevel boundary sensing RUNet segmentation algorithm.

**Figure 3:** (a) The original lung MRI image. (b) The segmented image of the lung nodules under the 3D U-Net. (c, d) The lung nodule segmented images under the multilevel boundary sensing RUNet, after the first and secondary segmentations, respectively.

**Figure 4:** Results of true positive, false positive, false negative, and Jaccard similarity of benign and malignant tumors.

**Figure 5:** Results of accuracy, sensitivity, and specificity of benign and malignant tumors.

**Figure 6:** Comparison of serum biochemical indicators between patients with benign and malignant lung tumors. ∗ indicates that the comparative differences were statistically significant (*P* < 0.05).

## Data Availability

The data used to support the findings of this study are available from the corresponding author upon request.
